The article "Anti-Inflammatory and Repairing Effects of Mesoporous Silica-Loaded Metronidazole Composite Hydrogel on Human Dental Pulp Cells" was retracted in 2023. Reasons: signs of a paper mill; suspected computer-generated content; unreliable results or conclusions; lack of ethics approval or compliance.

# Anti-Inflammatory and Repairing Effects of Mesoporous Silica-Loaded Metronidazole Composite Hydrogel on Human Dental Pulp Cells

**DOI:** 10.1155/2022/6774075

**Published:** 2022-03-23

**Authors:** Wei Wang, Xixi Wang, Luyang Li, Ying Liu

**Affiliations:** ^1^Oral Medical Center, Shenzhen People's Hospital (The Second Clinical Medical College, Jinan University, The First Affiliated Hospital, Southern University of Science and Technology), Shenzhen 518020, China; ^2^Department of Stomatology, The Affiliated Jiangning Hospital of Nanjing Medical University, Nanjing 211100, China

## Abstract

In order to test an effective biopolymer scaffold in promoting the growth of human dental pulp stem cells (HDPSCs), mesoporous silica @ hydrogel (MSN@Gel) nanocomposites are invented as a new type of biopolymer scaffold for HDPSCs proliferation in this paper. The expression levels of alkaline phosphatase (ALP), dentin matrix protein 1 (DMP1), and dentin sialophosphoprotein (DSPP) are significantly increased in the MSN@Gel group so as to better repair damaged dentin. In order to inhibit the proliferation of bacteria in the dental pulp, metronidazole (MTR) is loaded into MSN. The study found that MSN could effectively prolong the half-life of MTR by 1.75 times, and the viability of HDPSCs could be better maintained in the MSN-MTR@Gel group so as to better promote its proliferation to repair pulpitis. However, with the increase of the MTR concentration, its proliferation effect on HDPSCs decreased gradually, and the proliferation effect is the best in 10 *μ*mol/L. Therefore, the MSN-MTR@Gel scaffold is expected to become an effective method for pulpitis therapy in the future.

## 1. Introduction

Due to inadequate oral hygiene, wrong brushing methods, and bad eating habits, the incidence of pulpitis caused by dental caries is increasing year by year, and most of them are young patients. At present, root canal therapy is commonly used in pulpitis therapy. Although it can effectively remove the infection focus and control pain symptoms, adverse events may cause in permanent teeth whose root tips are not fully developed, such as root fracture and development stagnation [1, 2]. Therefore, it is a hot spot to improve the treatment of pulpitis in clinical research so as to get better treatment effect. The restoration of the tooth tissue in pulpitis is mainly to maintain the activity of the dental pulp and promote dentin regeneration. Good extracellular matrix (ECM) is needed to maintain the activity of human dental pulp stem cells (HDPSCs) so as to provide a scaffold for their growth, attachment, and differentiation [3]. At the same time, as a variety of pathogenic microorganisms exist in the oral cavity, infection is very easy to occur. Although mild inflammatory reaction can stimulate the proliferation and repair of HDPSCs, irreversible damage will be caused to HDPSCs if the inflammatory reaction is aggravated [4]. Therefore, it is necessary to continuously control the concentration of anti-inflammatory drugs in the process of dental pulp repair. The restoration of dentin is an important part in the process of dental pulp restoration. In the process of differentiation and restoration of HDPSCs, effectively improving its mineralization ability is an important condition to promote dentin restoration [5]. Relevant research shows that the harder ECM can make the cytoskeleton structure arranged more closely and orderly, which is conducive to cell mineralization [6]. Therefore, in the process of dental pulp repair, providing ECM with three-dimensional structure and strong mechanical properties is of great significance to improve HDPSCs activity and mineralization. With the development of tissue engineering technology, a variety of biological scaffolds of DPSCs have been successfully synthesized, which provides a good carrier for the regeneration and repair of dental pulp tissue.

The article "Anti-Inflammatory and Repairing Effects of Mesoporous Silica-Loaded Metronidazole Composite Hydrogel on Human Dental Pulp Cells" was retracted in 2023. Reasons: signs of a paper mill; suspected computer-generated content; unreliable results or conclusions; lack of ethics approval or compliance.

In this study, we chose hydrogel (Gel) as scaffold material for HDPSCs regeneration. Gel has a three-dimensional network structure similar to ECM and has good biocompatibility in vivo [7], which can mimic the microenvironment of DPSCs and regulate their growth. At the same time, in the process of dental pulp injury repair, the scaffold material needs to be filled in the root canal cavity, which is narrow and small. In order to effectively fill the cavity and provide a better microenvironment for HDPSCs' growth, the scaffold material needs to have good plasticity, and Gel has good fluidity and can effectively fill the pulp cavity [8]. However, the mechanical properties of the Gel is relatively poor, and it is difficult to support the adhesion and growth of HDPSCs, which will have adverse effects on the orderly arrangement of HDPSCs and further affect their mineralization ability [9]. Therefore, improving the mechanical properties of Gel is an urgent problem in clinical research. With the development of tissue engineering, many kinds of high strength Gels have been developed, such as double-network Gels and polymer cross-linked microsphere Gels [10]. However, their synthetic steps are complicated, which affect their clinical applications. With the development of nanotechnology, it provides new ideas for improving the mechanical properties of Gels. The crosslinking of inorganic nanoparticles (NPs) with Gel can form a Gel network, which can significantly improve Gel's mechanical properties [11], and the synthesis process is relatively convenient. In addition, the good drug loading ability of NPs can maintain the stable release of anti-inflammatory drugs in nanocomposite Gel so as to control the degree of inflammatory reaction effectively, which can better promote the adhesion and growth of HDPSCs.

The article "Anti-Inflammatory and Repairing Effects of Mesoporous Silica-Loaded Metronidazole Composite Hydrogel on Human Dental Pulp Cells" was retracted in 2023. Reasons: signs of a paper mill; suspected computer-generated content; unreliable results or conclusions; lack of ethics approval or compliance.

In this study, mesoporous silica NPs (MSNs) are selected as nanomaterials combined with Gels. MSN has good biocompatibility in vivo, and its pore size of surface pore structure can be customized according to actual requirements, thus controlling the release efficiency of drugs [12]. Otherwise, the inner part of MSN can provide larger space for drug loading [13]. At the same time, the modification of its surface can give it a variety of different functions, which is more conducive to its physiological role in vivo [14]. As a commonly used oral anti-inflammatory drug, metronidazole (MTR) has a good inactivation effect on bacteria in the oral cavity. Relevant studies show that sustained and mild inflammatory stimulation can better promote HDPSCs' proliferation and repair. MSN loaded MTR NPs can better control the release of MTR so as to maintain its concentration in Gels and provide a more stable microenvironment for HDPSCs' proliferation. Therefore, the antibacterial activity of MSN-loaded MTR composite Gel and its effect on HDPSCs' proliferation are discussed in this research.

## 2. The Preparation and Physicochemical Property Test

### 2.1. The Synthesis of MSN

250 mg hexadecyltrimethylammonium bromide (CTAB) (H5882-100G, Sigma-Aldrich, St. Louis, MO, USA) and 3 mL NaOH are dissolved in 120 mL dH_2_O. After stirring at 80 °C for 15 min, 1.3 g tetraethyl orthosilicate (TEOS) (333859-25 ML, Sigma-Aldrich) and 2.5 g ethanol are added to the above mixture. After stirring for 1 h, the supernatant is removed by centrifugation, and the precipitate is washed repeatedly with water. Then, the above particles are placed in 50 mL acid methanol all night to remove CTAB, and the centrifuged precipitate is cleaned with methanol and ethanol. Eventually, MSN is obtained by vacuum drying. In the later stage, MSN with and without MTR could be prepared.

### 2.2. The Synthesis of Gel and MSN@Gel Scaffold

500 mg sodium hyaluronate, 995 mg 1-ethyl-3-(3 (dimethylamino)propyl)carbodiimide (EDC) (MP4202-5G, Shanghai Jiqi Biotechnology Co., Ltd., China), and 576 mg *N*-hydroxysuccinimide (NHS) (130672-5G, Sigma-Aldrich) are dissolved in 100 mL dH_2_O at 26°C under magnetic stir for 1 h to form Gel; then, 25% MSN-MTR or MSN by total volume is added in Gel and composed MSN-MTR@Gel or MSN@Gel composite scaffold for standby.  Figure 1 shows the schematic of the assembly process for MSN-MTR@Gel and its mechanism.

The article "Anti-Inflammatory and Repairing Effects of Mesoporous Silica-Loaded Metronidazole Composite Hydrogel on Human Dental Pulp Cells" was retracted in 2023. Reasons: signs of a paper mill; suspected computer-generated content; unreliable results or conclusions; lack of ethics approval or compliance.

### 2.3. Detection of MTR Half-Life

The length of half-life has a key impact on drug dosage and efficacy. For the half-time test, MTR and MSN-MTR are administered intraperitoneally in C57BL/6 mice with a similar body weight of about 30 g. Blood samples are taken from the tail vein of the above-injected mice per hour, and the MTR concentration is detected for the half-time test.

## 3. The Proposed Method

### 3.1. Cell Culture of HDPSCs

HDPSCs (CP–H231, Procell, Wuhan, China) are cultured to assess the proliferation of MSN-MTR@Gel nanocomposites. These cells are cultured in 24-well plates for 24 h with HDPSCs complete culture medium (CM-H231, Procell) in a cell incubator (51032124, Thermo Fisher, MA, USA) under 37 °C and 5% CO_2_. Then, these cells are collected and diluted with PBS solution at a concentration of 1 × 10^4^ cells/mL for standby.

### 3.2. Adsorption of MSN@Gel Scaffold on HDPSCs

The MSN@Gel prepared in Section 2.1 is divided into three groups, 1 ml HDPSCs diluent prepared in Section 2.2 are inoculated on their surfaces, and then, 2 ml HDPSCs complete culture medium is added. The above HDPSCs are cultured in the cell incubator for 24 h. At 0, 12, and 24 h, the cultured HDPSCs are taken out, fixed with formaldehyde, and labeled with FITC staining. Then, the penetration of HDPSCs in the Gel is observed by using a confocal microscope (FV3000, OLYMPUS, Japan), and the scanning layer thickness is 50 *μ*m.

### 3.3. Detection of Mineralized Matrix Secreted by HPDSCs

The diluted HDPSCs prepared in Section 2.2 are divided into the control group, Gel group, and MSN-MTR@Gel group, and mineralization-inducing medium and HDPSCs complete culture medium are added into each group. Among which, HDPSCs are inoculated in the surface of Gel and MSN-MTR@Gel in the Gel group and MSN-MTR@Gel group, respectively. After cultured in a cell incubator for 14 days, 200 *μ*L Triton X-100 (X-100, Sigma-Aldrich, USA) is added to the cultured cells, and conventional PCR is used to detect the expression of ALP, DMP1, and DSPP in the lysed cell solution. The primer information is shown in Table 1.

### 3.4. Bacteria Culture and Live/Dead Test

*E. faecalis* (ATCC29212, Guangdong Huankai Microbial Technology Co., Ltd., China) and *S. mutans* (XYSW-JZ-1270, Shanghai Jiya Biotechnology Co., Ltd., China) represented the common streptococcus in the oral cavity and are used to detect antibacterial properties of MSN-MTR@Gel nanocomposites. *E. faecalis* and *S. mutans* are cultured in a 24-well plate for 8 h with glucose meat extract broth medium (LA3850, Solarbio, Beijing, China) in a microorganism incubator (51028133, Thermo Fisher, USA), and the growth conditions are 37 °C and 5% CO_2_. The cultured bacteria are adjusted to the concentration of 1 × 10^6^ CFU/mL and are divided into the Gel group and MSN-MTR@Gel Group, which are cultured in Gel and MSN-MTR@Gel, respectively. The activation state of *E. faecalis* and *S. mutans* is tested by using a live/dead bacterial kit (AAT-B22411, AAT Bioquest, USA). In this kit, MycoLight520 solution and propidium iodide solution are used to label live and dead bacteria, separately, and the released fluorescence is green and red.

The article "Anti-Inflammatory and Repairing Effects of Mesoporous Silica-Loaded Metronidazole Composite Hydrogel on Human Dental Pulp Cells" was retracted in 2023. Reasons: signs of a paper mill; suspected computer-generated content; unreliable results or conclusions; lack of ethics approval or compliance.

### 3.5. Activity Detection of HDPSCs under Different MTR Concentrations

The diluted HDPSCs prepared in Section 2.2 are divided into 3 groups. 1 mL MTR with concentrations of 1, 10, and 100 *μ*mol/L and 2 mL HDPSCs complete culture medium are added to the three groups, respectively. The above cells are cultured for 24 h in cell incubator under 37 °C and 5% CO_2_. The activity of HDPSCs in three groups is detected by immunofluorescence at 1 d, 7 d, and 14 d after culture. Anti-Ki-67 (ab15580, Abcam, USA) is used to label the active cells, and anti-caspase-3 (ab32351, Abcam) is used to mark apoptotic cells in each group. A confocal microscope is used to observe the fluorescence intensity.

### 3.6. Activity and Apoptosis Detection of HDPSCs In Vitro

To further evaluate the effect of Gel and MSN-MTR@Gel on the proliferation of HDPSCs, the diluted HDPSCs prepared in Section 2.2 are divided into the control group, Gel group, and MSN-MTR@Gel group, and HDPSCs are inoculated in the surface of Gel and MSN- MTR@Gel in the Gel group and MSN-MTR@Gel group, respectively. After added 2 mL HDPSCs complete culture medium, the above cells are cultured for 24 h in a cell incubator. The growth of cells is observed by an electron microscope (Axio Lab.A1, Beijing Pratt Instruments Co., Ltd., China), and the activity and apoptosis of HDPSCs in each group are detected by the same method in Section 2.6.

## 4. The Clinical Results

### 4.1. Characteristics of MSN-MTR@Gel Nanocomposite

In the process of differentiation repair, HDPSCs migrate from the pulp center to the surrounding damaged dentin, which is of great significance to reduce the repair time and promote the recovery. If MSN-MTR@Gel can guide HDPSCs to migrate internally, it will contribute to pulp repair from inside to outside. It is found that after cultured for 24 h, the fluorescence intensity of HDPSCs in each layer is different by scanning layer by layer through a confocal microscope, and the fluorescence intensity is the highest at the depth of 90 *μ*m, as shown in Figure 2(a). It indicated that the MSN-MTR@Gel could provide a good scaffold for HDPSCs' proliferation and guide them to migrate internally so as to better repair the damaged dentin. Otherwise, HDPSCs' mineralization ability is of great significance for dentin repair, and the high mechanical properties of ECM help HDPSCs to be more orderly arranged so as to improve the mineralization ability. It is found that compared with HDPSCs cultured in Gel, those cultured in the MSN-MTR@Gel arranged more orderly, adhered more closely, and had higher proliferation density, as shown in Figure 2(b), which is helpful for HDPSCs to better secrete mineralized matrix. In addition, the study found that the MSN-MTR could effectively prolong the half-life of MTR by 1.75 times, as shown in Figure 2(c), which could further reduce the dosage of MTR and improve its utilization.

The article "Anti-Inflammatory and Repairing Effects of Mesoporous Silica-Loaded Metronidazole Composite Hydrogel on Human Dental Pulp Cells" was retracted in 2023. Reasons: signs of a paper mill; suspected computer-generated content; unreliable results or conclusions; lack of ethics approval or compliance.

### 4.2. Mineralization Ability Detection of HDPSCs in Three Groups

The restoration of dentin is closely related to the mineralization ability of HDPSCs, and HDPSCs' mineralization ability is closely related to the mechanical properties of its growing ECM. The study found that compared with the control group, the expression of mineralization related factors is higher in Gel and MSN-MTR@Gel, such as ALP, DMP1, and DSPP, especially in the MSN-MTR@Gel group, as shown in Figure 3. It is suggested that the three-dimensional structure of the Gel provided a good scaffold for HDPSCs' proliferation and differentiation, and the addition of MSN-MTR further improved the mechanical properties of Gel, to better induce HDPSCs' mineralization ability.

### 4.3. Bacteriostatic Evaluation of MTR and MSN-MTR@Gel In Vitro

Due to the retention of food residues in the oral cavity, it is easy to breed bacteria, which is easily to cause pulpitis. In this study, *E. faecalis* and *S. mutans* are selected to explore the antibacterial properties of the Gel and MSN-MTR@Gel. As shown as Figure 4, the MSN-MTR@Gel could better inhibit the proliferation of the above bacteria, and more apoptotic bacteria are found. It indicated that Gel could act as antibacterial biofilms, and MSN drug delivery system could release MTR more effectively and enhanced its antibacterial properties.

### 4.4. HDPSCs Activity and Apoptosis Evaluation in Three Groups

The activity of HDPSCs in the repair process is of great significance to improve the efficiency and success rate of pulpitis therapy. In this study, we used Ki-67 to detect HDPSCs' activity. The study found that compared with the control group, the activity of HDPSCs cultured in Gel and MSN-MTR@Gel is higher, especially in the MSN-MRT@Gel Group, as shown in Figures 5(a), 5(b), and 5(c). In addition, caspase-3 is used to detect HDPSCs' apoptosis. It is found that compared with the control group, fewer apoptotic HDPSCs are found in Gel and MSN-MTR@Gel, especially in the MSN-MTR@Gel group, as shown in Figures 5(d), 5(e), and 5(f). The above results indicated that the Gel provided a good scaffold for HDPSCs' proliferation, and the addition of MSN-MTR could effectively control the growth of bacteria, to better improve the proliferative activity of HDPSCs and inhibit their apoptosis.

The article "Anti-Inflammatory and Repairing Effects of Mesoporous Silica-Loaded Metronidazole Composite Hydrogel on Human Dental Pulp Cells" was retracted in 2023. Reasons: signs of a paper mill; suspected computer-generated content; unreliable results or conclusions; lack of ethics approval or compliance.

### 4.5. Proliferation Detection of Different Concentrations of MTR on HDPSCs

The existence of anti-inflammatory drugs can control the number of bacteria and provide a good microenvironment for HDPSCs' proliferation. If the concentration of anti-inflammatory drugs is too high, its toxic and side effects will cause adverse effects on cell proliferation. We chose MTR's safe and effective drug concentration from 1 to 100 *μ*mol/L for study. It is found that when MTR's concentration is 10 *μ*mol/L, it had the best effect on HDPSCs' proliferation at the 7th and 14th day, and with the continuous increase of MTR's concentration, its proliferation effect is gradually weakened.  Figure 6 is proliferation detection of HDPSCs.

## 5. Clinical Result Analysis

As a common clinical disease in stomatology, the pain, oral inflammation, and other problems caused by pulpitis will seriously affect patients' life quality [15]. In pulpitis therapy, HDPSCs' activity is closely related to the self-healing ability of tooth tissue injury. On the one hand, maintaining HDPSCs' good activity is conducive to the self-repair of tooth tissue after inflammation control [16]. On the other hand, it is conducive to promote the later repair of dentin by inducing HDPSCs' mineralization. At present, how to effectively maintain pulp activity is a hot topic in clinical research. With the development of biotechnology, more and more new materials are used to maintain pulp activity, such as Gel, which has good histocompatibility and natural ECM structure. Therefore, if injected into the dental pulp cavity, Gel can fully wrap the irregular dental pulp cavity and encapsulate the dental pulp so as to support the migration and proliferation of HDPSCs [17]. As a result, the Gel is expected to become a new method for the therapy of pulpitis.

The Gel has good fluidity and plasticity so as to integrate with the irregular dental pulp cavity when injected into the endodontic cavity [18]. Secondly, the Gel has a three-dimensional structure similar to ECM, which provides a good scaffold for the adhesion and proliferation of HDPSCs so as to better enhance the contact and signal exchange between cells and improve HDPSCs' differentiation potential [19]. Thirdly, thanks to the good water retention ability of the Gel, it can enhance cell viability and reduce the occurrence of apoptosis events, and its good biocompatibility with the body can effectively reduce the inflammatory reaction [20]. In order to further improve HDPSCs' differentiation potential and promote the restoration of dentin, improving Gel's mechanical properties has a significant effect on HDPSCs' differentiation [21]. In this study, we combined MSN with Gel to prepare nanocomposites, thus significantly improving Gel's mechanical properties. At the same time, as a good drug carrier, MSN could better improve the bioavailability of loaded drugs [22]. It is found that MSN could increase the half-life of MTR by 1.75 times so as to reduce MTR's dosage and reduce its toxic and side effects while maintaining MTR concentration stably. Therefore, it is of great significance to study the repair effect of the MSN-MTR@Gel composite stent on dental pulp injury so as to improve the curative effect of pulpitis.

The article "Anti-Inflammatory and Repairing Effects of Mesoporous Silica-Loaded Metronidazole Composite Hydrogel on Human Dental Pulp Cells" was retracted in 2023. Reasons: signs of a paper mill; suspected computer-generated content; unreliable results or conclusions; lack of ethics approval or compliance.

In the process of pulpitis therapy, the migration of HDPSCs to the damaged tooth tissue is of great significance to improve the curative effect of pulpitis. In the study of Gel's adsorption properties, HDPSCs are found in different depths of Gel, and the fluorescence intensity is the highest at the depth of 60–90 *μ*m, suggesting that Gel has the potential of inducing and attracting HDPSCs. This is closely related to the three-dimensional structure of Gel, and its network structure can better promote HDPSCs adhesion and migration, thus more effectively repairing dental tissue. As the main component of dental hard tissue, the good repair of dentin is conducive to the protection of dental pulp so as to better promote the recovery of pulpitis. Dentin is secreted and synthesized by dentin cells. Therefore, inducing HDPSCs to differentiate into dentin cells and improving their mineralization ability are the key points in pulpitis therapy. It is found that the higher mechanical properties of the MSN-MTR@Gel complex could make the arrangement of HDPSCs more orderly and adhere more closely, thereby promoting HDPSCs' mineralization ability. As a result, the expression of ALP, DSPP, and DMP1 increases significantly in HDPSCs cultured in MSN-MTR@Gel, which can further promote the formation of dentin, thereby better protecting pulp and repairing damaged dental hard tissues.

Due to the deposition of food residues in the oral cavity, it is easy to be complicated with bacterial infection. In the process of dental pulp repair, controlling the inflammatory reaction in dental pulp cavity and inhibiting the release of inflammatory factors play a key role in maintaining the activity of dental pulp and reducing the damage of dental tissue. It is found that the MSN-MTR@Gel complex could better inhibit the proliferation of *E. faecalis* and *S. mutans*, thus inhibiting the invasion of the dental pulp cavity by oral bacteria, which is important for maintaining HDPSCs' activity and maintaining their physiological functions. MTR can effectively inactivate anaerobic bacteria in oral cavity, which plays an important role in maintaining HDPSCs' activity. However, with the increase of MTR concentration, its biosafety will also be adversely affected. It is found that when MTR's concentration is 1–100 *μ*mol/L, it could effectively promote HDPSCs' proliferation, and its proliferation effect is the best at 10 *μ*mol/L. Considering that at this concentration, it can better inhibit the concentration level of bacteria in pulp cavity, and mild inflammatory stimulation can better promote HDPSCs' proliferation. In addition, we found that compared with the control group, MSN-MTR@Gel complex and Gel could better maintain HDPSCs' activity and inhibit their apoptosis, especially in the MSN-MTR@Gel group, thus better promoting the repair of tooth damaged tissue.

The article "Anti-Inflammatory and Repairing Effects of Mesoporous Silica-Loaded Metronidazole Composite Hydrogel on Human Dental Pulp Cells" was retracted in 2023. Reasons: signs of a paper mill; suspected computer-generated content; unreliable results or conclusions; lack of ethics approval or compliance.

## 6. Conclusion

In this paper, we design a new biopolymer scaffold consisting of Gel and MSN. This paper finds that Gel promoted the migration of HDPSCs and could serve as a non-cell matrix scaffold for HDPSCs regeneration. At the same time, in order to inhibit bacteria's proliferation in the dental pulp, we loaded MTR with MSN. It is found that MSN could effectively increase the half-life of MTR by 1.75 times, and it could further improve the inhibition of Gel complex on *Streptococcus*, thereby reducing the inflammatory reaction and better maintaining the pulp activity. However, with the increase of MTR concentration, its proliferation effect on HDPSCs gradually decreased, and the proliferation effect is the best at 10 *μ*mol/L. Therefore, the MSN-MTR@Gel scaffold is expected to become an effective method for pulpitis therapy in the future.

## Figures and Tables

**Figure 1:** Schematic of the assembly process for MSN-MTR@Gel and its mechanism.

**Figure 2:** Physicochemical property test of the MSN-MTR@Gel system. (a) Distribution of HDPSCs under a confocal microscope (the depth of each layer is 50 *μ*m). (b) The growth of HDPSCs in the Gel group and MSN@Gel group. (c) Half-life period test of MSN-MTR and purely MTR injection.

**Figure 3:** Detection of mineralization ability of HDPSCs. (a) ALP expression level in HDPSCs. (b) DMP1 expression level in HDPSCs. (c) DSPP expression level in HDPSCs. ^*∗∗∗*^*P* < 0.001.

**Figure 4:** Growth of *E. faecalis* and *S*. *mutans* on Gel. (a) Live staining of cultured *E*. *faecalis* 8 h after adding Gel. (b) Live staining of cultured *E*. *faecalis* 8 h after adding MSN-MTR@Gel. (c) Dead staining of cultured *E*. *faecalis* 8 h after adding Gel. (d) Dead staining of cultured *E*. *faecalis* 8 h after adding MSN-MTR@Gel. (e) Live staining of cultured *S. mutans* 8 h after adding Gel. (f) Live staining of cultured *S. mutans* 8 h after adding MSN-MTR@Gel. (g) Dead staining of cultured S mutans 8 h after adding Gel. (h) Dead staining of cultured *S. mutans* 8 h after adding MSN-MTR@Gel.

The article "Anti-Inflammatory and Repairing Effects of Mesoporous Silica-Loaded Metronidazole Composite Hydrogel on Human Dental Pulp Cells" was retracted in 2023. Reasons: signs of a paper mill; suspected computer-generated content; unreliable results or conclusions; lack of ethics approval or compliance.

**Figure 5:** HDPSCs activity and apoptosis assessment. (a) Anti-Ki-67 expression pattern in the control group. (b) Anti-Ki-67 expression pattern in the Gel group. (c) Anti-Ki67 expression pattern in the MSN-MTR@Gel group. (d) Anti-caspase-3 expression pattern in the control group. (e) Anti-caspase-3 expression pattern in the Gel group. (f) Anti-caspase-3 expression pattern in the MSN-MTR@Gel group.

**Figure 6:** Proliferation detection of HDPSCs. (a–c) Proliferation of HDPSCs in MTR with the concentration of 1 *μ*mol/L at 1 d, 7 d, and 14 d. (d–f) Proliferation of HDPSCs in MTR with the concentration of 10 *μ*mol/L at 1 d, 7 d, and 14 d. (g–i) Proliferation of HDPSCs in MTR with the concentration of 100 *μ*mol/L at 1 d, 7 d, and 14 d.

**Table 1:** Primer information of PCR.

	F primer	R primer
ALP	5′-ATGGGATGGGTGTCTCCACA-3′	5′-CCACGAAGGGGAACTTGTC-3′
DMP1	5′-ATATTGAGGGCTGGAATGGGGA-3′	5′-TTTGTGGCTCCAGCATTGTCA-3′
DSPP	5′-TGGAGCCACAAACAGAAGCAA-3′	5′-TCCAGCTACTTGAGGTCCATC-3′
GAPDH	5′-TCACCATCTTCCAGGAGCGAGAC-3′	5′-AGACACCAGTAGACTCCACGACATAC-3′

## Data Availability

The simulation experiment data used to support the findings of this study are available from the corresponding author upon request.
